The article "Characteristics of lumbar scoliosis in patients with rheumatoid arthritis" was published in 2014. Journal: J Orthop Surg Res.

# Characteristics of lumbar scoliosis in patients with rheumatoid arthritis

**DOI:** 10.1186/1749-799X-9-30

**Published:** 2014-04-26

**Authors:** Masanobu Ohishi, Hisaaki Miyahara, Masakazu Kondo, Yasuharu Nakashima, Kazumasa Terada, Yukio Esaki, Nobuo Kobara, Katsumi Harimaya, Yoshihiro Matsumoto, Yukihide Iwamoto

**Affiliations:** 1 Department of Orthopaedic Surgery, Faculty of Medical Sciences, Graduate School of Medicine, Kyushu University, 3-1-1 Maidashi Higashiku, Fukuoka 812-8582, Japan; 2 Department of Orthopaedic Surgery and Rheumatology, Clinical Research Institute, National Hospital Organization Kyushu Medical Center, Fukuoka 810-8563, Japan; 3 Kondo Clinic of Rheumatology and Orthopaedics, Fukuoka 810-0001, Japan

**Keywords:** Rheumatoid arthritis, Scoliosis, Osteoporosis, Bisphosphonate

## Abstract

**Background:**

Although a substantial percentage of patients with rheumatoid arthritis (RA) experience low back pain, the characteristics of lumbar spine pathology in RA patients has been poorly investigated. In our institutions, lumbar spine radiographs indicated scoliosis in 26 patients. The present study aimed to clarify the characteristics of lumbar scoliosis in RA patients.

**Methods:**

This is a retrospective study of 26 RA patients with lumbar scoliosis. Patient characteristics such as disease duration, disease stage and class according to Steinbrocker's classification, and medication for RA and osteoporosis were reviewed. Radiologic evaluation of scoliosis was performed at two different time points by measuring Cobb angles. The progression of scoliosis per year was calculated by dividing the change in Cobb angles by the number of years. Apical vertebral rotation, lateral listhesis, and the level of the intercrestal line at the first observation were also measured. The correlation between different factors and changes in the Cobb angles per year was analyzed.

**Results:**

Majority of the patients had a long disease duration and were classified as stage 3 or 4 according to Steinbrocker's classification. During the observation period, most patients were treated with glucocorticoids. Unlike the previous studies on degenerative scoliosis, apical vertebral rotation, lateral listhesis, and the level of the intercrestal line at initial observation were not significantly related to the progression of scoliosis. Initial Cobb angles were inversely related to the progression of scoliosis. Patients who were treated with bisphosphonates showed slower progression of scoliosis.

**Conclusions:**

Our results indicate that the characteristics of lumbar scoliosis in RA patients differ from those of degenerative lumbar scoliosis. Bone fragility due to the long disease duration, poor control of disease activity, and osteoporosis is possibly related to its progression.

## Background

Rheumatoid arthritis (RA) is an inflammatory disorder that affects multiple joints. In addition to the joints of the extremities, the atlantoaxial ligament of the cervical spine is often affected by synovial inflammation. Thus, the involvement of the cervical spine in RA has been studied extensively [1]. In contrast, the pathology of the thoracic and lumbar spine in RA patients has been poorly studied. More than 30%–50% of RA patients reportedly experience back pain and have a higher degree of disability and depression than those without back pain [2-4]. Therefore, clarifying the characteristics of lumbar spine pathology in RA patients is clinically highly relevant. In 1964, Lawrence et al. [5] found an increased incidence of subluxation, disc narrowing, apophyseal destruction, and osteoporosis of the lumbar spine in RA patients compared with that in non-RA controls. Based on these criteria, they estimated that rheumatoid changes were present in the lumbar spines of 3%–5% of RA patients. In our medical institutions, we found that the radiographs of RA patients indicated scoliosis, which was defined as a lateral curvature of the spine >10°. We performed a retrospective study of 26 RA patients who presented with lumbar scoliosis. By evaluating the radiographic findings and the backgrounds of these patients, we attempted to determine the pathological characteristics of this condition.

## Materials and methods

This retrospective case series included 26 patients with RA who presented at the National Kyushu Medical Center, Kyushu University Hospital, or Kondo Clinic of Rheumatology. The institutional review boards approved the study. The most recent radiographs of these RA patients indicated lumbar scoliosis with a Cobb angle of ≥10°. Cobb angles in the first and most recent radiographs were measured using supine anteroposterior images. The changes in the Cobb angles were divided by the number of years between two time points to evaluate the yearly progression. Apical vertebral rotation was measured according to the criteria introduced by Nash and Moe [6]. Lateral listhesis and the level of the intercrestal line were measured as documented elsewhere [7]. Patient characteristics such as age, sex, and disease duration were reviewed. To evaluate disease control during the observation period, both disease stage and class according to Steinbrocker's classification [8] were assessed. Medications for both RA and osteoporosis were reviewed. The destruction of the hip and knee joints was evaluated using the Larsen method [9]. For statistical analyses, Mann-Whitney *U* test or ANOVA was performed. Mann-Whitney *U* test was used for the comparison of the data between two groups, and ANOVA was used for the comparison of the data between three groups or more. *P* < 0.05 was accepted as significant.

## Results

Baseline characteristics of the 26 patients are summarized in Table 1. Mean disease duration was 21.8 years, and 24 patients had disease duration >10 years. According to Steinbrocker's classification, most patients had advanced stage (stage 3 and stage 4) RA (Table 1). The disease-modifying antirheumatic drugs that the patients were taking were methotrexate, sulfasalazine, bucillamine, and biologic agents. Importantly, all but one patient were taking a glucocorticoid (Figure 1).

**Table 1:** Clinical features of 26 patients with scoliosis

	**Value**
Age, years (average ± SD)	54 ~ 84 (70.16 ± 9.14)
Sex	
Female	22
Male	4
Disease duration, years (average ± SD)	4 ~ 46 (21.8 ± 10.3)
Steibrocker's classification	
Stage 2	2
Stage 3	6
Stage 4	18
Class 1	3
Class 2	18
Class 3	4
Class 4	1

**Figure 1:** **Disease-modifying antirheumatic drugs used for the treatment of 26 RA patients.** The percentage of the patients using each drug is shown. *SASP/BCL* salazosulfapyridine or bucillamine, *MTX* methotrexate, *Bio* biologic agents.

The mean Cobb angle at the initial observation was 17.18° ± 9.29°, which progressed to 24.5° ± 10.2° within a mean 4.32 years (Figure 2). The mean change in the Cobb angle per year was 1.80°.

**Figure 2:** **Progression of scoliosis.** Year 0 indicates the first observation time point.

Regression analysis between yearly changes in Cobb angles and initial Cobb angles showed that the scoliosis of those with larger initial Cobb angles progressed more slowly (Figure 3). There was a correlation between the two values (*r* = −0.505). Those with apical vertebral rotation ≥ grade 2 tended to show faster progression of scoliosis, although the difference was not statistically significant (Figure 4). Neither lateral listhesis nor the level of the intercrestal line was correlated with the progression of scoliosis (data not shown). The majority of our patients showed erosive changes around the endplates, whereas proliferative changes were not so evident (Figure 5). We next investigated the osteoporosis management of our patients. As shown in Figure 6A, 7 of 26 patients did not receive osteoporosis treatment. The remaining patients received bisphosphonate (BP) with or without a vitamin D (VitD) analog (15 patients), only a VitD analog (3 patients), or a selective estrogen receptor modulator (SERM) (1 patient) (Figure 6A). The progression of scoliosis calculated by the yearly change in the Cobb angle was 0.70° in the BP treatment group, 3.94° in the VitD treatment group, 1.5° in the SERM treatment group, and 3.28° in the no treatment group. Interestingly, when the patients were divided into those who were treated with and without BP, the former showed significantly slower progression of scoliosis than the latter (Figure 6B).

**Figure 3:** Regression analysis of Cobb angle at initial observation and change in Cobb angle per year.

**Figure 4:** **The relationship between grade of apical vertebral rotation and change in Cobb angle per year.** Error bars represent means ± SEM.

**Figure 5:** **This patient is a 70-year-old woman with RA and scoliosis with a 24-year history of RA.** Progression of scoliosis and changes of radiological findings were evaluated between 2005 and 2008. The radiographs taken in 2005 (*left panels*) and 2008 (*right panels*) are shown. The *lines* in the anteroposterior views (*upper panels*) indicate the upper and lower tilting vertebrae. The *arrows* of both anteroposterior and lateral (*lower panels*) views indicate progression of disc space narrowing and endplate destruction.

**Figure 6:** **Treatment of osteoporosis and progression of scoliosis. (A)** The progression of scoliosis in each osteoporosis treatment group is shown. **(B)** Comparison of scoliosis progression between those who were treated with BP and those who were not. *Error bars* represent means ± SEM. *Tx* treatment, *VitD* vitamin D analog, *BP* bisphosphonates, *SERM* selective estrogen receptor modulator.

To determine whether the hip and/or knee joint status affects the progression of scoliosis, we divided the patients into three groups based on the severity of the hip and knee joints affected. Group A included those who underwent joint replacement or joint damage of Larsen grade 3/4 of the hips and/or knees of the bilateral limbs. Group B included those with joint replacement or joint damage of Larsen grade 3/4 of the unilateral lower limbs. In group A, five patients underwent bilateral total hip and/or knee replacement, and in group B, six patients underwent unilateral total hip and/or knee replacement. One patient in group B had unilateral knee joint damage of Larsen grade 4, and 14 had no joint damage greater than Larsen grade 2 and were categorized as group C. The progression of scoliosis tended to be faster in group A than in the other groups, although the difference was not statistically significant (data not shown).

## Discussion

In this study, we investigated the characteristics of lumbar scoliosis in RA patients. Previous studies have shown that a larger initial Cobb angle, a higher grade of apical vertebral rotation, a greater degree of lateral listhesis, and the intercrestal line through or below the L4/5 disc space are predictors of the progression of degenerative scoliosis [7,10]. In the present study, the initial Cobb angle was inversely related to the yearly increase in the Cobb angle, which is contrary to what has been reported for degenerative scoliosis. Other factors did not show a statistically significant relationship with scoliosis progression. These findings suggested that other factors might be involved in the progression of scoliosis in RA patients.

Bone fragility is a typical pathological feature of RA [11]. Although the present study lacks bone mineral density data, the scoliosis itself would make accurate measurement difficult. The majority of our patients were already at either stage 3 or stage 4 according to Steinbrocker's classification after a long disease duration, which indicates poor disease control in those patients. Furthermore, all but one patient were taking a daily dose of a glucocorticoid. Thus, it is presumable that the bones of those patients were fragile, and we hypothesize that bone fragility is part of the pathogenesis of scoliosis in RA patients. It has been reported by Mawatari et al. [12] that RA patients can lose substantial vertebral strength after a mean of 12.2 months. Of note, the bone strength of the patients treated with alendronate was significantly higher than that in those who did not receive antiresorptive treatment. It is quite intriguing that, in our study, patients who were treated with BPs showed significantly slower progression of scoliosis than those who were not treated with BPs, which indicates that BP administration was, at least in part, protective against the progression of scoliosis. Recent studies have shown that BP is effective for the management of glucocorticoid-induced osteoporosis in terms of fracture prevention [13,14], which has been reflected in the treatment guidelines for this condition in different countries [15,16]. Thus, our data reconfirmed the importance of BP treatment from a perspective different from fracture prevention.

In 25 of our patients, we observed erosive changes around the endplates, which is a typical finding of the rheumatoid spine [17-21]. With respect to the erosive changes of the endplates, two different theories have been proposed. One is the involvement of an inflammatory response in the disc lesion. This theory is supported by the observation that inflammatory tissue in the rheumatoid thoracic spine appeared to originate in the costovertebral articulations and extended into the nearby discovertebral junction [20]. The other theory is that discovertebral alterations are related to traumatic events produced by instability in the posterior elements of the spine. According to the radiographic-pathologic correlative study by Schils et al. [18], no evidence of synovial infiltration was observed in the disc lesion. A similar result was reported also by Martel [19], who found reactive fibrosis but no inflammation in the destructive lesion of the discovertebral junction of the cervical spine. Magnetic resonance images of 13 of our patients did not show any obvious signal change of the facet joints or the endplates, and currently, we do not have evidence that our patients had facet joint or endplate inflammation (data not shown).

Disability of the lower extremities, especially the hip joints, is known to influence lumbar spine degeneration, which has been documented as hip-spine syndrome [22]. Because RA patients often develop severe hip and/or knee joint deformity, the effect of both hip and knee joint destruction on scoliosis progression was studied. Those who underwent bilateral hip/knee joint replacement showed a tendency to progress faster than those who did not, although the difference was not statistically significant. Furthermore, because the progression of scoliosis in those who underwent unilateral total joint replacement or had severe joint damage of the lower limb was not affected, the limb length discrepancy *per se* would not be related to the progression.

The limitation of the present study is that the number of patients studied is too small to perform multivariate analysis. However, scoliosis in RA patients itself is not a major entity, and it will be extremely difficult to accumulate a large number of patients. Although we used supine anteroposterior radiographs, standing radiographs, which are standard for the evaluation of scoliosis, would have shown even more severe deformity. Moreover, in terms of studying the factors affecting the progression speed of scoliosis, we believe that our data are still valuable because the radiographs were taken under the same conditions.

## Conclusions

Our data indicate that the characteristics of the progression of scoliosis in RA patients differ from those of degenerative scoliosis. Bone fragility resulting from the disease activity of RA and glucocorticoid treatment is possibly related to its progression.

## Competing interests

MO received speaking fees from Chugai Pharmaceutical, Ono Pharmaceutical, Pfizer, Eisai, and Eli Lilly. HM received speaking fees from Chugai Pharmaceutical, Takeda Pharmaceutical, Mitsubishi-Tanabe Pharma, Janssen Pharmaceutical, Pfizer, Eisai, Abbott, and Bristol-Myers. MK received speaking fees from Chugai Pharmaceutical, Takeda Pharmaceutical, Mitsubishi-Tanabe Pharma, Janssen Pharmaceutical, Pfizer, Eisai, Abbott, and Bristol-Myers. YN received speaking fees from Chugai Pharmaceutical, Mitsubishi-Tanabe Pharma, and Abbott. YI received speaking fees from Chugai Pharmaceutical, Takeda Pharmaceutical, Mitsubishi-Tanabe Pharma, Janssen Pharmaceutical, Pfizer, Eisai, and Abbott. All fees were less than US$5,000 each. All other authors declare that they have no competing interests.

## Authors' contributions

MO, HM, and MK conceived of the study. MO carried out the data collection and performed the statistical analysis and drafted the manuscript. MK, KT, YE, NK, and YN also carried out the data collection. KH, YM, and YI participated in the design and coordination and helped draft the manuscript. All authors read and approved the final manuscript.
